# Histone deacetylase inhibitors reduce differentiating osteoblast-mediated protection of acute myeloid leukemia cells from cytarabine

**DOI:** 10.18632/oncotarget.21809

**Published:** 2017-10-10

**Authors:** Rosalie M. Sterner, Kimberly N. Kremer, Aref Al-Kali, Mrinal M. Patnaik, Naseema Gangat, Mark R. Litzow, Scott H. Kaufmann, Jennifer J. Westendorf, Andre J. van Wijnen, Karen E. Hedin

**Affiliations:** ^1^ Mayo Clinic Medical Scientist Training Program, Mayo Clinic College of Medicine and Science, Rochester, Minnesota 55905, USA; ^2^ Department of Immunology, Mayo Clinic College of Medicine and Science, Rochester, Minnesota 55905, USA; ^3^ Division of Hematology and Department of Medicine, Mayo Clinic College of Medicine and Science, Rochester, Minnesota 55905, USA; ^4^ Department of Oncology, Mayo Clinic College of Medicine and Science, Rochester, Minnesota 55905, USA; ^5^ Department of Orthopedic Surgery and Department of Biochemistry and Molecular Biology, Mayo Clinic College of Medicine and Science, Rochester, Minnesota 55905, USA

**Keywords:** AML, osteoblast, HDACi, vorinostat, panobinostat

## Abstract

The bone marrow microenvironment protects acute myeloid leukemia (AML) cells during chemotherapy and is a major factor in relapse. Here, we examined which type(s) of bone marrow cells are responsible for the relapse of AML following treatment with cytarabine (Ara-C), and we identified a means to inhibit this protection. To determine the protective cell type(s), AML cells were treated with Ara-C, and AML cell survival in the presence or absence of osteoblast lineage cells was assessed. Cultured AML cells and patient bone marrow isolates were each significantly protected from Ara-C-induced apoptosis by co-culture with differentiating osteoblasts. Moreover, pretreating differentiating osteoblasts with the histone deacetylase inhibitors (HDACi) vorinostat and panobinostat abrogated the ability of the differentiating osteoblasts to protect AML cells. Together, our results indicate that differentiating osteoblasts have the potential to promote residual AML in the bone marrow following standard chemotherapy and act via a mechanism requiring HDACi-sensitive gene expression. Using HDACi to target the leukemic microenvironment in combination with Ara-C could potentially improve treatment of AML. Moreover, other strategies for manipulating bone marrow osteoblasts may also help eradicate AML cells and reduce relapse.

## INTRODUCTION

Despite the high initial remission rates achieved with the chemotherapeutic cytarabine (Ara-C) for acute myeloid leukemia (AML), chemoresistance and subsequent relapse of disease are common [1–4]. Identifying and targeting the mechanisms that mediate the chemoresistance of this residual disease will be critical to enhancing the efficacy of Ara-C treatment for AML.

Residual AML cells are located in the bone marrow microenvironment [1, 2]. *In vivo* animal studies have identified the endosteal region (tissue between the bone marrow and ossified surface) of the bone marrow as the location of Ara-C-resistant AML cells [5, 6]. Osteoblast lineage cells of the endosteal region promote the survival of various cell types [7–12]. This lineage begins with bone marrow mesenchymal stromal/stem cells that give rise to osteoprogenitors that develop into osteoblasts and then osteocytes [13, 14]. In particular, osteoblasts have been described as protectors of AML cells to both daunorubicin- and SDF-1-induced apoptosis [15–17]. Therefore, identifying the specific cell type(s) that provide protection to AML cells from Ara-C-induced apoptosis may provide a means to target chemoresistance.

AML is one of many malignancies for which histone deacetylase inhibitors (HDACi) are being investigated, and HDACi have shown initial promise in combination therapies with Ara-C [18–24]. HDACi prevent deacetylation of multiple proteins including histones and leave chromatin in a more open configuration, provoking widespread changes in gene expression. While HDACi, such as vorinostat (suberoylanilide hydroxamic acid; SAHA) and panobinostat (LBH589), are capable of directly altering gene expression within malignant cells, HDACi also alter gene expression of osteoblast-lineage cells [25–28]. Modulation of osteoblast-lineage cell functions may explain why HDACi have shown limited efficacy alone but more promise in combination with standard chemotherapeutics [18–24].

Here, we characterize differentiating osteoblasts as potent protectors of AML cells from Ara-C-induced apoptosis using a co-culture model. In addition, we identify HDACi as a means to disrupt chemoresistance by targeting osteoblast-mediated protection of AML cells. Together, these results suggest that manipulating the protective cells within the bone marrow may be an effective strategy for enhanced sensitization of AML cells to standard chemotherapy, improved AML cell eradication, and prevention of relapse.

## RESULTS

### Differentiating MC3T3 osteoblasts protect KG1a AML cells from Ara-C-induced apoptosis

Normal and leukemic hematopoiesis is supported by osteoblasts [8, 15, 29]. In addition, we previously showed that differentiating osteoblasts protect AML cell lines and patient isolates from SDF-1, a chemokine that is abundant in the bone marrow yet induces AML cell apoptosis [16, 17, 30]. If differentiating osteoblasts protect AML cells from SDF-1-induced apoptosis, we hypothesized that they may also protect AML cells from Ara-C and induce chemoresistance. To test this idea, we utilized our previously described co-culture model that combines the KG1a AML cell line with the well-characterized, rapidly mineralizing MC3T3 sc4 osteoblast cell line (Figure 1A). Osteogenic differentiation of MC3T3 cells was initiated on Day 0 upon addition of osteogenic medium. After 2 days (a time point we previously showed was sufficient for MC3T3 cells to acquire the ability to protect AML cells from SDF-1-induced apoptosis) [16], KG1a cells were added to MC3T3 cell cultures for 1 hour, followed by the indicated dose of Ara-C, and the co-cultures were incubated for an additional 16-18 hours. Apoptosis was then assayed via flow cytometric detection of annexin-V binding. Figure 1B shows representative results; Figures 1C, 1D summarize the results of multiple independent experiments. As expected, addition of Ara-C increased the percentage of annexin-V positive KG1a cells in a dose-dependent manner over a range of 0.5 μM-10 μM. Co-culture with differentiating MC3T3 cells significantly decreased the percentage of annexin-V positive KG1a cells even at the highest dose of 10 μM Ara-C. To ensure that Ara-C was not simply killing the MC3T3 cells, live/dead assays were conducted to assess MC3T3 viability. Even at the highest dose of Ara-C (10 μM), no significant increase in MC3T3 cell death was detectable compared to vehicle-treated MC3T3 cells (∼2% dead cells) (Figure 1E). Thus, differentiating MC3T3 osteoblasts protect co-cultured AML cells from Ara-C-induced apoptosis.

**Figure 1:** Differentiating MC3T3 osteoblasts protect KG1a AML cells from Ara-C-induced apoptosis **(A)** Diagram illustrating the KG1a AML cell line-MC3T3 osteoblast co-culture model. On day 0, osteogenic differentiation medium was added to MC3T3 cells. On day 2, MC3T3 cells were rinsed with PBS, KG1a cells were then added, and cells were treated with either vehicle (PBS) or the indicated concentration of Ara-C. On day 3, KG1a cell apoptosis was assayed via annexin-V staining and flow cytometry. **(B)** Results of a representative experiment performed as in A, showing the % of apoptotic annexin-V positive KG1a cells from each culture. **(C)** Summary of multiple experiments performed as in A and B using 1 μM Ara-C; bars depict mean apoptosis of KG1a AML cells ± S.E.M., *n=3*; ^*^, significantly different from control (*p*≤0.05). **(D)** Summary of multiple experiments performed as in A-C using 0 μM (PBS, indicated as 10^-8^ on dose curve), 0.1 μM, 0.5 μM, 1 μM, 5 μM, and 10 μM doses of Ara-C; each point depicts mean apoptosis of KG1a AML cells ± S.E.M., *n=3*; ^*^, *p*≤0.05. **(E)** Assay to ensure MC3T3 cell viability in the presence of Ara-C during co-culture. Experiments were performed as in A except that no KG1a cells were added. Confocal microscopy and live/dead staining was used to reveal live (green) and dead (red) cells in MC3T3 monolayers. Images were acquired on 3 separate days for a total of 15 images per condition.

### Differentiating MC3T3 osteoblasts protect patient AML isolates from Ara-C

We next investigated whether MC3T3 osteoblasts could protect primary AML cells from Ara-C induced apoptosis. AML patient isolates were cultured either with or without differentiating MC3T3 cells, challenged with either Ara-C or vehicle, and analyzed for apoptosis. Consistent with the results observed in the AML cell line, MC3T3 co-culture consistently protected AML cells, even in the presence of Ara-C (Figure 2A-2D). The average fold change in the percentage of annexin-V positive AML patient cells induced by 1 μM Ara-C was decreased by MC3T3 co-culture for the four AML patient bone marrow isolates examined (Figure 2C). Moreover, the decrease was significant: MC3T3 co-culture consistently reduced AML cell apoptosis by approximately 5-fold in the presence of 1 μM Ara-C (Figure 2C). Together with data in Figure 1, these results indicate that osteoblasts can protect co-cultured AML cells from Ara-C-induced apoptosis.

**Figure 2:** Differentiating MC3T3 osteoblasts protect patient AML isolates from Ara-C **(A)** Diagnostic bone marrow aspirates were obtained from different AML patients prior to chemotherapy and combined with differentiating MC3T3 osteoblast monolayers. After 1 hour of co-culture, cells were challenged with 0 μM (PBS, indicated as 10^-8^ on dose curve), 0.05 μM, 0.1 μM, 0.2 μM, 0.5 μM, 1 μM, 5 μM, and 10 μM doses of Ara-C. After 48-72 hours, patient AML cells were assayed for apoptosis via annexin-V staining and flow cytometry as in Figure 1. The dose curve for patient 30 is depicted in A. **(B)** Clinical AML samples from four patients performed as in A using PBS or 1μM Ara-C. **(C)** Summary of results from analyzing patient samples as in A and B showing the average fold change in apoptotic annexin-V positive AML cells in response to 1 μM Ara-C in either the absence or presence of MC3T3 cells. Bars depict mean results ± S.E.M. for four different patients; ^*^, significantly different from cultures lacking MC3T3 cells (*p*≤0.05). **(D)** Patient information. “Positive” represents the presence of an activating mutation (internal tandem duplication or Asp-835 mutations), and “negative” represents the lack of an activating mutation.

### An immortalized human BMSC cell line fails to protect KG1a AML cells from Ara-C-induced-apoptosis

To determine whether the protective properties of osteoblasts are generalizable to other bone marrow cells of the osteoblast-lineage, we tested bone marrow-derived mesenchymal stromal/stem cells (BMSC), a developmental precursor to osteoblasts, for their ability to protect KG1a cells from Ara-C. The KG1a cell line was cultured either alone or with a confluent layer of a human bone marrow-derived tert-immortalized BMSC cell line in the presence of vehicle or Ara-C and subsequently assayed for apoptosis (Figure 3A). In contrast to differentiating MC3T3 osteoblasts (Figures 1-2), BMSC provided no significant protection to the AML cells across the entire dose range of 0.1 μM-10 μM Ara-C (Figure 3B-3D). In fact, co-culturing with BMSC slightly increased the apoptosis of KG1a AML cells in response to 10 μM Ara-C (Figure 3D). Ara-C was not simply killing the BMSC cells since live/dead viability assays showed that vehicle and 10 μM Ara-C treatment each resulted in approximately 0.4% and 0.3%, respectively, of dead (red) cells and a predominately live (green) monolayer of cells (Figure 3E). These results indicate that BMSCs (developmental precursors of osteoblasts) do not protect AML cells from Ara-C, in contrast to differentiating osteoblasts.

**Figure 3:** An immortalized human BMSC cell line fails to protect KG1a AML cells from Ara-C-induced-apoptosis **(A)** Diagram illustrating the KG1a AML cell line-BMSC co-culture model. On day -1, BMSC cells were plated. On day 2, KG1a AML cells were added to confluent BMSC monolayers, and cultures were challenged with either vehicle (PBS) or the indicated concentration of Ara-C. On day 3, the apoptosis of KG1a cells was assayed via annexin-V staining and flow cytometry as in Figure 1. **(B)** Results of a representative experiment performed as in A, showing the % of annexin-V positive KG1a cells from each culture. **(C)** Summary of multiple experiments performed as in A and B using 1 μM Ara-C; bars depict mean results ± S.E.M., *n=3*; ^*^, significantly different from control (*p*≤0.05). **(D)** Summary of multiple experiments performed as in A-C using the indicated doses of Ara-C; each point depicts mean apoptotic KG1a cells ± S.E.M., *n=3*; ^*^, *p*≤0.05. **(E)** BMSC cell viability was assayed as in Figure 1E on 3 independent days for a total of 15 images for each condition.

### Vorinostat pre-treatment of differentiating MC3T3 osteoblasts reduces osteoblast-mediated protection of KG1a AML cells from Ara-C-induced apoptosis

We next tested whether we could diminish osteoblast-mediated protection of AML cells from Ara-C by using HDACi to alter osteoblast gene expression patterns. Day 1 differentiating MC3T3 osteoblasts were pretreated with vehicle or the HDACi vorinostat or panobinostat for 30 hours. At the end of this preincubation, the HDACi was removed, osteoblasts were washed, KG1a cells were added, and co-cultures were treated with vehicle or Ara-C for 16-18 hours before annexin-V binding was assessed (Figure 4A). Vorinostat treatment increased acetylation of Histone H3 in differentiating MC3T3 cells as expected (Figure 4B). Interestingly, vorinostat pre-treated MC3T3 cells exhibited a significant reduction in their ability to protect KG1a AML cells from Ara-C-induced apoptosis compared to vehicle-treated MC3T3 cells (Figure 4C and 4D). We previously reported that vorinostat slightly increased the percentage of dead (red) MC3T3 cells (∼6%) compared to DMSO (∼1%); however, vorinostat-treated MC3T3 cells still formed a confluent monolayer of predominantly live (green) cells [30]. Thus, the differentiating osteoblast-mediated protection of AML cells from Ara-C can be reduced via the HDACi vorinostat.

**Figure 4:** Vorinostat pre-treatment of differentiating MC3T3 osteoblasts reduces osteoblast-mediated protection of KG1a AML cells from Ara-C-induced-apoptosis **(A)** Diagram illustrating the KG1a AML cell line-MC3T3 co-culture model used to analyze vorinostat pretreatment of MC3T3. On day 0, osteogenic differentiation media was added to MC3T3 cells. On day 1, either 0.1% DMSO, 10 μM vorinostat, or 1 μM panobinostat was added to the MC3T3 cells. On day 2, MC3T3 cells were rinsed to remove vorinostat or panobinostat, then KG1a cells were added, and cultures were treated with either vehicle (PBS) or the indicated concentration of Ara-C. On day 3, the apoptosis of KG1a cells was assayed via annexin-V staining and flow cytometry as in Figure 1. **(B)** Immunoblot confirming the effect of vorinostat on MC3T3 cells. MC3T3 cells cultured as in A were harvested on day 2 and whole cell lysates immunoblotted to reveal acetylation of Histone H3 (Ac-H3) in response to vorinostat treatment. The same membrane was stripped and re-blotted for total histone-3 as a control, *n*=3. **(C)** Summary of multiple experiments performed as in A using 1 μM Ara-C; bars depict mean results ± S.E.M., *n=3*; ^*^, significantly different from control (*p*≤0.05). **(D)** Summary of multiple experiments performed as in A-C using the indicated doses of Ara-C; each point depicts mean apoptosis of KG1a AML cells ± S.E.M., n=3. ^*^, results from vorinostat + MC3T3 co-cultures were significantly different from results from vehicle (DMSO) + MC3T3 co-cultures, *p*≤0.05.

### Panobinostat pre-treatment of differentiating MC3T3 osteoblasts inhibits osteoblast-mediated protection of KG1a AML cells from Ara-C-induced apoptosis

Because we had observed reduction in differentiating osteoblast-mediated protection from Ara-C in AML cells with vorinostat pre-treatment of differentiating MC3T3 cells, we hypothesized that we would see similar effects using a second HDACi, panobinostat, if this reduction of protection was indeed induced via a HDACi sensitive mechanism. The expected increase in acetylation of Histone H3 in differentiating MC3T3 cells was observed with panobinostat treatment (Figure 5A). Panobinostat pretreatment of differentiating MC3T3 cells inhibited their ability to protect KG1a AML cells from Ara-C-induced apoptosis compared to differentiating MC3T3 cells pre-treated with vehicle (Figure 5B). Interestingly, panobinostat pre-treatment of differentiating MC3T3 cells also resulted in increased AML cell apoptosis even without treatment with Ara-C compared to AML cells that were not treated with Ara-C and were not co-cultured with differentiating MC3T3 cells (Figure 5B). Panobinostat only slightly increased the percentage of dead (red) MC3T3 cells (∼3%) compared to DMSO (∼0.7%), and panobinostat-treated MC3T3 cells still formed a confluent monolayer of predominantly live (green) cells. Together, the results show that differentiating osteoblasts, but not their BMSC precursors, potently inhibit the Ara-C-induced apoptosis of co-cultured AML cells via a mechanism sensitive to HDACi (Figure 6).

**Figure 5:** Panobinostat pre-treatment of differentiating MC3T3 osteoblasts inhibits osteoblast-mediated protection of KG1a AML cells from Ara-C-induced-apoptosis **(A)** Immunoblot confirming the effect of panobinostat on MC3T3 cells. MC3T3 cells were cultured and immunoblotted for acetylation of Histone H3 (Ac-H3) and Histone H3 as in Figure 4B, *n*=4. **(B)** Summary of multiple experiments performed as in Figure 4A using 1 μM Ara-C; bars depict mean results ± S.E.M., *n=4*; ^*^, results from panobinostat + MC3T3 co-cultures were significantly different from results from vehicle (DMSO) + MC3T3 co-cultures, *p*≤0.05. **(C)** MC3T3 cell viability was assayed as in Figure 1E on 4 independent days for a total of 20 images for each condition (0.1% DMSO or 1 μM panobinostat treatment with experiments performed as in Figure 4A except cells underwent imaging on day 2 instead of KG1a cells and Ara-C being added).

**Figure 6:** Model of AML cell protection from Ara-C-induced apoptosis by differentiating osteoblasts within the endosteal niche of the bone marrow **(A)** Based on results in this paper, we propose that differentiating osteoblasts within the endosteal niche of the bone marrow are likely responsible for protecting nearby AML cells from Ara-C-induced apoptosis. **(B)** Our results presented here additionally indicate that pretreating differentiating osteoblasts with the HDACi vorinostat or panobinostat substantially inhibit their ability to protect AML cells from Ara-C.

## DISCUSSION

Unfortunately, a small population of AML cells that reside in the bone marrow is resistant to the chemotherapeutic Ara-C and often leads to relapse, suggesting that the bone marrow may contribute to the chemoresistance of these residual cells [1–3]. Osteoblast lineage cells within the endosteal region of the bone marrow possess the ability to promote the survival of hematopoietic stem cells (HSC) and various leukemic cells [7-9, 11, 12]. Thus, it is possible that osteoblast lineage cells induce phenotypic changes of the AML cells that reside in the endosteum that permit the AML cells to become chemoresistant. Identifying the specific cell type of the bone marrow microenvironment that protects AML cells and targeting the protective mechanisms may lead to more effective combination treatments with Ara-C. Here, we not only identify differentiating osteoblasts as potent protectors of AML cells but also report a strategy to inhibit this protection.

We utilized a well-characterized co-culture system [16, 30] that permits assessment of the ability of osteoblast lineage cells to protect AML cells from Ara-C-induced apoptosis and also permits manipulation of the osteoblast lineage cells to identify means of blocking the protection. We show that differentiating MC3T3 osteoblasts potently and consistently protected KG1a AML cells from Ara-C-induced apoptosis. Additionally, differentiating osteoblasts protected all co-cultured primary AML isolates examined to date even in the presence of Ara-C. These results are consistent with the linkage of an increase in osteoblast-secreted factors with both worse prognosis and the development of chemoresistance in AML [15, 31]. In contrast, stromal cells from various species and organs have been described to both enhance and inhibit survival of AML cells in response to various apoptosis-inducing agents [12, 16, 32, 33]. Interestingly, AML patient-derived BMSC were able to protect AML cells while healthy donor-derived BMSC were not [12]. These contradictory results may be due to the source of stromal cells or the possibility that leukemic cells influence the BMSC to acquire osteoblast characteristics. Here, we showed that a tert-immortalized BMSC human cell line failed to block Ara-C-induced apoptosis in KG1a AML cells, despite the ability of these BMSC to promote the survival of hematopoetic stem cells and acute lymphoblastic leukemia (ALL) cells in studies by others [7, 34]. Together, these results suggest that differentiating osteoblasts could contribute to the chemoresistance of the residual AML cells found in the endosteal niche following Ara-C treatment.

We next sought to identify a means to manipulate the bone marrow microenvironment in order to prevent AML cell resistance to Ara-C. Though HDACi are capable of directly altering gene expression within malignant cells, they are also known to alter gene expression of osteoblast lineage cells [25–28]. We report here that pretreating osteoblasts with the HDACi vorinostat or panobinostat was sufficient to prevent their protection of AML cells from Ara-C-induced apoptosis. This is consistent with our previous observation that vorinostat or panobinostat pre-treatment of osteoblasts inhibited their ability to protect AML cells from SDF-1-induced apoptosis via activation of a Nherf1-PP1a-TAZ signaling pathway [30]. This pathway led to the nuclear localization of TAZ, a transcription factor that regulates osteoblast differentiation via regulation of osteogenic genes [35–37]. These results and the observation that HDACi can alter gene expression of osteoblast-lineage cells *in vitro* may help explain the increased efficacy seen in clinical trials combining HDACi with Ara-C compared to either treatment alone [18–24].

To our knowledge, this is the first study to suggest that differentiating osteoblasts could play a critical role in the development of AML cell resistance to Ara-C. Although osteoblasts have been shown to mediate HSC and leukemic cell survival [7-9, 11, 12], the mechanism(s) by which osteoblasts induce chemoresistance of AML cells is not well-characterized. Daunorubicin-induced death of the U937 AML cell line was partially inhibited by osteoblasts via the Wnt antagonist sFRP-1 [15]. In addition, SDF-1-induced apoptosis was inhibited by differentiating osteoblasts in a cell contact-independent manner [16], suggesting that protection is mediated via a soluble factor. These results demonstrate that osteoblasts protect AML cells from various apoptosis-inducing agents, despite the distinct mechanisms utilized by daunorubicin, SDF-1, and Ara-C to induce apoptosis. Further experimentation will be necessary to determine if osteoblasts utilize a universal mode of protection or a distinct mode of protection for each apoptosis-inducing agent.

In summary, our results reported here identify differentiating osteoblasts within the bone marrow microenvironment as potent protectors of AML cells from apoptosis induced by the standard chemotherapeutic Ara-C. Moreover, we have also identified a means to disrupt this protection via the HDACi vorinostat and panobinostat. HDACi may therefore be effective in combination with Ara-C as an improved treatment for AML. Further characterization and targeting of the molecular mechanisms utilized by osteoblasts to protect AML cells could provide additional, more specific means to prevent chemoresistance and relapse.

## MATERIALS AND METHODS

### Materials

Ascorbic acid, β-glycerophosphate, dimethylsulfoxide, protease inhibitor cocktail, and Ara-C were purchased from Sigma (St. Louis, MO, USA). Vorinostat was obtained from the Cancer Therapy Evaluation Program, National Cancer Institute (Bethesda, MD, USA). Panobinostat was purchased from Selleckchem (Houston, TX, USA). Live/dead viability assays were purchased from Invitrogen (Waltham, MA, USA). Anti-acetylated Histone H3 and Anti-total Histone H3 were purchased from Millipore (Darmstadt, Germany).

### Cells

After obtaining informed consent, bone marrow samples were harvested from AML patients prior to chemotherapy according to an IRB-approved protocol. After sedimentation on a Ficoll-Paque (1.077 g/cm^3^) step gradient [38], recovered mononuclear cells were cultured in Medium A as described [16]. The KG1a human AML cell line (ATCC, Manassas, VA, USA) was cultured as described [16]. The human bone marrow-derived tert-immortalized BMSC cell line (BMSC) was derived from primary mesenchymal cells from unfractionated bone marrow mononuclear cells transduced with hTERT (gift from Dario Campana, St. Jude, Memphis, TN, USA) [34] and cultured as described [16]. MC3T3 sc4 murine calvarial osteoblasts were maintained in MC3T3 medium (α-MEM without ascorbic acid (Invitrogen, Carlsbad, VA, USA), 10% FCS, and 1% penicillin/streptomycin) [39]. Prior to use in assays, MC3T3 cells were plated in 12-well plates and upon reaching confluence were treated (day 0) with osteogenic differentiation medium (α-MEM, 10% FCS (v/v), 1% penicillin/streptomycin (v/v), 50 μg/ml ascorbic acid, and 4 mM β-glycerophosphate).

### Co-cultures, HDACi treatment, and apoptosis assay

On day minus 1, MC3T3 or BMSC cells were plated in 12 well plates in their respective maintenance media. On day 0, osteogenic differentiation medium was added to MC3T3 cells. On day 1, 0.1% DMSO or 10 μM vorinostat was added as indicated. Due to the short half-life of vorinostat [40, 41], the 10 μM vorinostat dose was selected to ensure persistent Histone H3-acetylation (a marker of vorinostat activity) within vorinostat-treated MC3T3 cells for the duration of the 30 hour pretreatment period [26, 30]. The 1 μM panobinostat dose exhibited persistent Histone H3-acetylation in panobinostat-treated MC3T3 cells for the duration of the 30 hour pretreatment period [30]. On day 2, the cells were rinsed with PBS, given fresh medium consisting of RPMI and 10% FCS, and 0.25 x 10^6^ cells/ml of KG1a cells were added to the co-cultures. After one hour, vehicle (PBS) or the indicated concentration of Ara-C was added to each well. On day 3, apoptosis of KG1a cells was assayed via APC-conjugated annexin-V staining to detect surface phosphatidylserine via flow cytometry. A two-tailed t-test was used for statistical analysis (Microsoft Excel) with the means of the two distributions being considered significantly different if *p* ≤0.05. For clinical AML isolates, AML cells were cultured in Medium A [16] for 1-2 hours prior to plating with MC3T3 cells. MC3T3 cells were cultured in osteogenic medium for 1-24 hours prior to co-culture with AML bone marrow aspirates. (For patient 30 only, 0.1% DMSO (in osteogenic medium) was added to MC3T3 cells for 2 hours prior to replacement with fresh osteogenic medium for an additional 1-2 hr.) 0.25 x 10^6^ cells/ml of primary AML cells were then added to wells with or without differentiating MC3T3 cells, co-cultured for 1 hour, and treated with either vehicle (PBS) or the indicated concentration of Ara-C for 48-72 hours prior to analysis of AML cell apoptosis.

### Live/dead cell viability assay

A LSM780 laser scanning confocal microscope (Carl Zeiss, Oberkochen, Germany) with ZEN software (Carl Zeiss), a 10X/0.45 M27 objective, and excitation/emission wavelengths of 561 nm/626 nm (dead; red) and 488 nm/522 nm (live; green) was used for these assays. The percentage of dead cells was determined by dividing the number of dead cells by the number of live plus dead cells.

## Abbreviations

AML: acute myeloid leukemia
HADCi: histone deacetylase inhibitors
BMSC: bone marrow-derived mesenchymal stromal/stem cells
v/v: volume/volume
